# Bioinformatics Analysis of Potential Biomarkers and Pathway Identification for Major Depressive Disorder

**DOI:** 10.1155/2021/3036741

**Published:** 2021-08-03

**Authors:** Dong Qi, Kui Chen

**Affiliations:** Beijing Friendship Hospital Affiliated to Capital Medical University, China

## Abstract

Aiming at a more comprehensive understanding of the molecular biomarkers and potential mechanisms of major depressive disorder (MDD), from the Gene Expression Omnibus (GEO) database, we first obtained mRNA expression profiles and identified 585 differentially expressed genes (DEGs) through the R software, including 263 upregulated genes and 322 downregulated genes. Then, through the Kyoto Encyclopedia of Genome and Genome (KEGG) pathway and biological process (BP) analysis, we found that the upregulated and downregulated DEGs were abundant in different pathways, respectively. It was noteworthy that upregulated DEGs were the most significantly enriched in the mTOR signaling pathway. Subsequently, through the protein-protein interaction (PPI) network, we identified seven hub genes, namely, EXOSC2, CAMK2A, PRIM1, SMC4, TYMS, CDK6, and RPA2. Finally, through gene set enrichment analysis (GSEA), we obtained that hypoxia, epithelial-mesenchymal transition, hedgehog signaling, and reactive oxygen species pathway were the enriched pathways for MDD patients. The above data results would provide a new direction for the treatment of MDD patients.

## 1. Introduction

Major depressive disorder (MDD) is a typical depressive disorder. The main clinical manifestations are marked by lasted depression and loss of interest [1]. In severe cases, psychiatric symptoms such as hallucinations and delusions may occur, accompanied by suicidal behavior [2]. At present, MDD has become a major human disease “killer” in the 21st century. More than millions of people die of the disease every year. Among them, 20-30 years old is the main age of onset, and female patients are more common than male [3]. And the data for 2020 also showed that MDD had become the second most common human disease after cardiovascular disease. Although the clinical cure rate of MDD is very high, the treatment rate and recurrence rate of the disease are not very optimistic because of patients' insufficient knowledge and unwillingness to regular treatment [4]. So far, the specific cause of MDD is still unclear. At present, it is only understood that the interaction of environmental, psychological, endocrine, and other factors has a paramount impact on the pathogenesis of MDD [5]. Therefore, the biomarkers that have a paramount impact on the pathogenesis of MDD still need further study.

There have been many research reports on the treatment of MDD. For example, the study by Fagiolini and Kupfer discusses the progress of MDD in diagnosis, neurobiology, and treatment. The results find that in nearly 40% of patients, major depression is related to life-long isolated manic or hypoglycemic symptoms [6]. Further research has been done on the specific psychotherapy for depression, the clinical application of antidepressants, the development of new therapeutic compounds, etc. Experiments by Jazvinscak Jembrek et al. show that the human intestinal flora may play a role in stress, anxiety, and depression. It also confirmed that there is two-way communication between the brain and the intestines [7]. Long-term use of probiotics is beneficial to alleviate anxiety and depression and other related behaviors, thereby helping to alleviate the distress of mental illnesses. Zhang et al. systematically evaluate the relationship between the tumor necrosis factor-*α*G-308A gene polymorphism and the risk of depression through meta-analysis and obtain the allele frequency of the tumor necrosis factor-*α*G-308A gene [8]. Neither gene type nor genotype can be used as an independent risk factor for depression, and further exploration is needed on the specific influencing factors of MDD.

The Gene Expression Omnibus (GEO) is a free high-throughput microarray and related functional genomic dataset [9]. In this study, mRNA expression profiles were downloaded based on the GEO database for analysis of the underlying mechanisms and biomarkers of MDD. 25 MDD samples and 25 normal samples were collected in the GSE54563 database. Through making use of the Limma package in the R software, we screened 585 differentially expressed genes (DEGs). These genes had the potential to be new diagnostic biomarkers. Through the Kyoto Encyclopedia of Genes and Genomes (KEGG) pathway [10], Gene Ontology (GO) analysis [11], and protein-protein interaction (PPI) network [12], the potential molecular mechanisms affecting MDD were analyzed. The seven hub genes were EXOSC2, CAMK2A, PRIM1, SMC4, TYMS, CDK6, and RPA2. Based on the above database, we could gain a more comprehensive understanding of MDD and obtain new therapeutic targets.

## 2. Materials and Methods

### 2.1. Microarray Data Archives

The expression configuration file of the GSE54563 (https://www.ncbi.nlm.nih.gov/geo/query/acc.cgi) array was retrieved based on the GEO database. The microarray dataset GSE54563 was deposited by Chang et al. The glutamate- and GABA-enriched gene module related to human depression was identified by coexpression meta-analysis and DNA variant genome-wide association studies. 50 total samples in 25 pairs were analyzed in postmortem tissue from the anterior cingulate cortex. The samples of the MDD group and control group were selected for further analysis. On the basis of the GPL6947 Illumina HumanHT-12 V3.0 Expression BeadChip, we finished the expression analysis of this database. From the GEO database, we downloaded the series of matrix files and data table header descriptions of GSE54563 aiming at screening and verifying the central genes involved in MDD.

### 2.2. Differentially Expressed Gene (DEG) Identification

The threshold criterion for DEG identification was *P* < 0.05 between MDD and control samples, according to the Limma package in R software. Then, we drew the heat map of DEGs through the Pheatmap package in R software.

### 2.3. GO and KEGG Pathway Enrichment Analyses

As a common tool used to analyze bioinformatics, Gene Ontology (GO) contains comprehensive functional information related to each gene. GO analysis includes three parts: cell component (CC), biological process (BP), and molecular function (MF). KEGG is a database that integrates chemistry, genome, and system function information aimed at understanding advanced biological functions and practicality. The GO annotation and KEGG pathway enrichment analyses of the identified DEGs were performed using DAVID 6.8 (https://david.ncifcrf.gov/). The results were considered statistically significant if *P* < 0.05.

### 2.4. PPI Network Creation and Hub Gene Identification

On the basis of the Search Tool for the Retrieval of Interacting Genes (STRING 11.0; https://string-db.org/), we constructed the PPI network, with a combined score > 0.4 as the cut-off point. We identified the hub genes by Cytoscape software 3.7.1 (https://www.cytoscape.org/).

### 2.5. Gene Set Enrichment Analysis

The related biological pathways in 25 MDD and 25 normal samples selected from the GSE54563 dataset were analyzed by GSEA (https://software.broadinstitute.org/gsea/index.jsp).

## 3. Results

### 3.1. Identification of DEGs Related to MDD

Aiming at identifying DEGs in MDD, we searched the relevant microarray expression profile of GSE54563 from the GEO database. As shown in the heat map, after the integration and standardization of the microarray data, we got 585 DEGs, which contained 263 upregulated DEGs and 322 downregulated DEGs (Figure 1).

### 3.2. KEGG Enrichment Analysis of DEGs

KEGG pathway analysis presented that upregulated DEGs were obviously abundant in signaling pathways regulating pluripotency of stem cells, mTOR signaling pathway, Hippo signaling pathway, RNA degradation, hepatocellular carcinoma, adrenergic signaling in cardiomyocytes, PI3K-Akt signaling pathway, and other pathways (Figure 2(a)). Downregulated DEGs were obviously abundant in small-cell lung cancer, chemical carcinogenesis, Fc gamma R-mediated phagocytosis, Fc epsilon RI signaling pathway, ether lipid metabolism, DNA replication, regulation of lipolysis in adipocytes, and other pathways (Figure 2(b)).

### 3.3. BP Enrichment Analysis of DEGs

On the basis of the DAVID online tool, the biological process GO terms of DEGs were analyzed. According to the results in Figure 3(a), for the upregulated DEGs, synapse assembly, neuron projection development, calcium ion transport into the cytosol, regulation of cardiac muscle cell apoptotic process, and canonical Wnt signaling pathway were significantly enriched terms. In addition, the downregulated DEGs were major abundant in gliogenesis, cellular response to osmotic stress, positive regulation of interleukin-1 beta production, myelination, regulation of oxidative stress-induced intrinsic apoptotic signaling pathway, and other pathways (Figure 3(b)).

### 3.4. PPI Network Analysis

DEGs' PPI network formed by STRING determined the important clusters of DEG. Among the PPI network of upregulated DEGs, there were 216 nodes and 167 edges. The significant pivot node genes were selected with degrees ≥ 5 as the screening criterion; among these genes, EXOSC2 had the highest node degree (degree = 9) and the degree of CAMK2A was top 2 (degrees = 7) (Figure 4). 270 nodes and 254 edges together formed a PPI network of downregulated DEGs (Figure 5). With degree ≥ 10 as the screening criterion, the top 5 significant genes were screened out as PRIM1, SMC4, TYMS, CDK6, and RPA2.

### 3.5. Identification of MDD-Associated Pathways

In order to further explore the key biological pathway associated with MDD, GSEA was used on the database GSE54563. Results revealed that the pathways of “hypoxia,” “epithelial-mesenchymal transition,” “hedgehog signaling,” and “reactive oxygen species” were enriched in MDD patients (Figure 6).

## 4. Discussion

MDD is the main type of mood disorder, the result of the interaction between physical, psychological, and social factors [13]. It usually manifests as depression, decreased volition, slow thinking, sleep disturbance, fatigue, loss of appetite, weight loss, constipation, pain in body parts, and other symptoms [14]. At present, mild depression is generally relieved through exercise first [15]. If not improved, antidepressant drugs and combined psychotherapy are taken later. As for severe depression, it may need a combination of antidepressants and antipsychotics, antidepressants, and psychotherapy or electroconvulsive therapy [16]. As for short-term treatment, benzodiazepines are recommended if the patient suffers from acute suicidal depression, catatonic depression, or depression with symptoms, such as insomnia and anxiety [17]. However, because MDD is a complex mental illness, most patients' understanding of the disease is still at the superficial stage, and they are even afraid of admitting or concealing the symptoms without cooperating with active treatment. In addition, the current clinic cannot provide individualized treatment based on the specific neurobiological mechanism of the patient. Therefore, this kind of disease is still seriously disturbing the daily life of patients. In this study, we analyzed the key genes in MDD through bioinformatics methods and tried to find effective biomarkers and potential therapeutic targets.

As for this research, through the R software, we found 585 DEGs in total, including 263 upregulated DEGs and 322 downregulated DEGs. On the basis of BP and KEGG analysis, upregulated DEGs were obviously abundant in synapse assembly, neuron projection development, mTOR signaling pathway, and other pathways. Downregulated DEGs were obviously abundant in gliogenesis, cellular response to osmotic stress, Fc epsilon RI signaling pathway, and other pathways. The report by Chandran et al. points out that by activating the mTOR signaling pathway in mammals, ketamine can produce a rapid antidepressant response [18]. Experiments in mice prove that p70S6K, mTOR, eIF4B, and p-eIF4B protein expressions in the control group are obviously higher than those in the MDD group. It also shows that mTOR-dependent translation initiation is defective in MDD, and there may be a correlation between the apparent lack of synaptic protein and the dysregulation of mTOR signaling in MDD [19]. Combined with our enrichment analysis results, we suggest that MDD is largely associated with the mTOR signaling pathway.

In addition, we also found that EXOSC2 and CAMK2A were hub upregulated genes and PRIM1, SMC4, TYMS, CDK6, and RPA2 were hub downregulated genes. The full name of EXOSC2 is exosome component 2. As a protein-coding gene, it is usually associated with short stature, hearing loss, retinitis pigmentosa, and type 1B pontine cerebellar hypoplasia [20]. Related pathways include CDK-mediated phosphorylation and removal of Cdc6 and ATP/ITP metabolism. CAMK2A belongs to the Ca (2^+^)/calmodulin-dependent protein kinase subfamily [21]. Calcium signaling has a vital impact on several aspects of glutamatergic synaptic plasticity [22]. The related pathways are the MAPK signaling pathway, oxidative stress pathway, and GPCR signaling. The GO annotations about this gene are inclusive of protein homopolymerization activity and protein kinase activity. PRIM1 is usually associated with Seckel syndrome and telangiectatic osteosarcoma disease. It is generally enriched in the synthesis of the telomere C chain (lagging chain) and the G1/S phase pathway of mitosis [23]. SMC4 belongs to the chromosome structure maintenance (SMC) gene family [24]. Members included in this gene family have a paramount impact on the chromosome structural changes during chromosome mitosis. SMC4 is the core of the clusterin complex necessary for chromosome assembly and separation. This gene is usually expressed in pleural empyema and Cornelia de Lange syndrome. And it is enriched in the pathway where activated PKN1 stimulates AR (androgen receptor) to regulate the transcription of genes KLK 2 and KLK 3 and metaphase. CDK6 belongs to the CMGC family of serine/threonine protein kinases [25]. The kinase is the catalytic subunit of the protein kinase complex and has a vital impact on the progression of the G1 phase of the cell cycle and the G1/S transition. The report by Diehl et al. confirms that CDK4 and CDK6 can assist cells to enter the S phase of the cell division cycle in the process of mammalian cell proliferation [26]. In the future, we can further explore the role of these genes in MDD.

Not only that, but also we performed GSEA analysis on GSE54563. The results indicated that MDD patients were significantly associated with hypoxia, epithelial-mesenchymal transition, hedgehog signaling, and reactive oxygen species pathway. Huang et al. pointed out in the study that ABL1 has abnormal regulation in both MDD and cancer depression patients. High levels of reactive oxygen species can cause ABL1 to activate oxidative stress and participate in MDD. The study by Myint et al. also confirmed that reactive oxygen species are related to the expression of MDD. Rana et al. discussed the role and potential of hedgehog signaling in the development of MDD and found that this pathway plays an important role in neurogenesis and neural tube formation and may be related to the pathogenesis of MDD.

This study has some limitations. First, our study was analyzed using public databases, but after screening the genes that are the key to MDD, the function of the key genes should be further explored through in vitro and in vivo experiments. Secondly, the expression levels of the key genes were not explored; their expression levels and mechanism of action will be explored in future studies.

In a word, 585 DEGs were identified related to MDD in this study, including 263 upregulated genes and 322 downregulated genes. Then, the potential mechanism of DEGs was determined through enrichment analysis. The upregulated DEGs are significantly enriched in the mTOR signaling pathway. Subsequently, the key genes of MDD were analyzed through PPI network analysis, including EXOSC2, CAMK2A, PRIM1, SMC4, TYMS, CDK6, and RPA2. Finally, the key pathways associated with MDD were obtained by GSEA. The analysis results show that hypoxia, epithelial-mesenchymal transition, hedgehog signaling, and reactive oxygen species pathways are the enrichment pathways of DEGs. We have discovered some important biological processes and pathways and the hub genes that play a role in these processes, providing new insights for the development and progression of MDD disease and providing methods for the subsequent treatment of MDD patients.

## Figures and Tables

**Figure 1:** Heat map of 585 DEGs which were screened using the R software Limma package. The red areas stand for upregulated genes, and the blue areas stand for downregulated genes. DEG: differentially expressed gene.

**Figure 2:** Enrichment analysis of upregulated (a) and downregulated (b) differential genes by KEGG pathways. KEGG: Kyoto Encyclopedia of Genes and Genomes.

**Figure 3:** Enrichment analysis of upregulated (a) and downregulated (b) differential genes by BP. BP: biological process.

**Figure 4:** PPI network of upregulated genes contains 216 nodes and 167 edges. PPI: protein-protein interaction. Nodes mean proteins, and edges mean the interaction of proteins.

**Figure 5:** PPI network of downregulated genes contains 270 nodes and 254 edges. PPI: protein-protein interaction. Node means proteins, and edges mean the interaction of proteins.

**Figure 6:** Gene set enrichment analysis (GSEA) in database GSE54563: (a) hypoxia; (b) epithelial-mesenchymal transition; (c) hedgehog signaling; (d) reactive oxygen species pathway.

## Data Availability

All data analyzed during this study were obtained from the published article or are available from the corresponding author on reasonable request.
